# LncRNA SNHG15 Promotes Oxidative Stress Damage to Regulate the Occurrence and Development of Cerebral Ischemia/Reperfusion Injury by Targeting the miR-141/SIRT1 Axis

**DOI:** 10.1155/2021/6577799

**Published:** 2021-11-26

**Authors:** Mingming Kang, Fangchao Ji, Xingyuan Sun, Hongbin Liu, Chenxin Zhang

**Affiliations:** ^1^Department of Neurology, The Third Affiliated Hospital of Qiqihar Medical University, Ward 3, Qiqihar 161000, China; ^2^President's Office, The Third Affiliated Hospital of Qiqihar Medical University, Qiqihar 161000, China

## Abstract

Ischemic stroke is a kind of disease with high mortality and high disability, which brings a huge burden to the public health system (Hu et al. (2017)), and it poses a serious threat to the quality of life of patients. Cerebral ischemia/reperfusion injury is an important pathophysiological mechanism. This study aims to assess the mechanism of SNHG15 in the occurrence and development of cerebral ischemia/reperfusion injury of nerve cells and to investigate its potential value for diagnosis and treatment. SNHG15 targeted miRNA molecules and target genes were predicted with bioinformatics tools such as StarBase and TargetScan. The process of ischemic reperfusion in cerebral apoplexy in normal cultured and oxygen-glucose-deprived and reoxygenated neurons was simulated with RT-PCR and western blot technique. The expressions of SNHG15 and miR-141 were detected with qPCR, and the expressions of SIRT1 and p65, TNF-*α*, ROS, iNOS, and IL-6 were detected with western blot. Meanwhile, SNHG15 siRNAs and miR-141 mimics were transfected for SH-SY5Y, with western blot testing. And the expressions of miR-141, SIRT1, and p65, TNF-*α*, ROS, iNOS, and IL-6 were tested. According to the prediction with bioinformatics tools of StarBase and TargetScan, miR-141 is the target of lncSNHG15. In the luciferase reporter plasmid double-luciferase assay, miR-141 and SIRT1 were defined as the target relationship. In the oxygen-glucose-deprived reoxygenation model group, SNHG15 expression increased, miR-141 expression decreased, SIRT1 expression increased, and the expressions of p65, TNF-*α*, ROS, iNOS, and IL-6 decreased. In the SNHG15-siRNA-transfected oxygen-glucose-deprived reoxygenation cell model group, miR-141 expression increased, SIRT1 expression decreased, and the expressions of p65, TNF-*α*, and IL-6 increased compared with the si-NC group. In the miR-141-mimic-transfected oxygen-glucose-deprived reoxygenation cell model, SNHG15 expression decreased, SIRT1 expression decreased, and the expressions of p65, TNF-*α*, IL-1*β*, and IL-6 increased. In conclusion, SNHG15 expression increased during the process of oxygen-glucose-deprived reoxygenation, and the oxidative stress process was reduced by miR-141/SIRT1.

## 1. Introduction

Ischemic stroke is a kind of disease with high mortality and high disability, which brings a huge burden to the public health system [1]. Cerebral ischemia/reperfusion injury (CIR) is a kind of neurological injury caused by ischemia and hypoxia after cerebral ischemia, which may lead to microvascular dysfunction or even aggravation of neurological injury when blood perfusion is restored in a short period of time. Therefore, we need to find safe and effective drugs to intervene in CIR, which may effectively improve the prognosis of patients. The oxygen-glucose-deprived (OGD) reoxygenation model can effectively simulate the pathophysiological process of brain CIR in vitro by simulating the glucose-free environment with a hypoxia device combined with a glucose-free medium. It was transferred to a normal oxygen concentration and glucose medium to continue culturing after treatment for a period of time as the pathophysiological process of CIR. SH-SY5Y cells are human neuroblastoma, which can be used in neuronal injury in vitro models because they are similar to neurons in morphology, neurochemistry, and electrophysiological characteristics. Therefore, OGD reoxygenation treatment on SH-SY5Y cells can be used as a recognized cell model in the study of CIR, so as to be widely used [2, 3].

Long noncoding RNAs (lncRNAs) are a set of noncoding RNAs of more than 200 nucleotides in length, which play an important role in transcription and translation, thus participating in regulating the mechanism of apoptotic oxidative stress neuroinflammation [4]. Several studies have confirmed that lncRNAs can play an important role in the pathophysiological mechanism of CIR [5]. LncRNAs, as competitive endogenous RNAs, can suppress miRNA functions through specific binding with microRNA (miRNA), thus regulating the expression of miRNA target genes [6]. After CIR, lncRNA H19 expression will increase to further promote the death of neurons by regulating miR-21 expression and initiating programmed necrosis of microglial cells [7]. Small nucleolar RNA host gene 14 (SNHG14) may contribute to the inflammatory response to CIR by regulating miR-136 expression, so as to aggravate its nerve injury [8]. After CIR, SNHG12 expression can increase and activate autophagy by regulating the functions of mesenchymal stem cells, thus increasing the death of neurons. Downregulation of SNHG12 expression can increase the functions of mesenchymal stem cells, reducing autophagy and apoptosis in cerebral microvascular endothelial cells, thus protecting the neurons [9].

Recent studies have observed the upregulation of small nucleolar RNA host gene 15 (SNHG15) expressions in cells treated with CIR. However, its specific mechanism is not clear [10]. The related studies of tumor series have shown that SNHG15 can specifically bind to miR-141 and act as endogenous RNA to regulate the expression of sirtuin 1 (SIRT1), the target gene of miR-141 [11]. And studies have observed that depressing miR-141 expression may relieve symptoms associated with ischemic stroke, but the pathophysiological mechanism remains unclear [12]. SIRT1 can regulate such pathophysiological processes as oxidative stress through deacetylated histone and related transcription factors, playing an important role in the pathophysiological process of myocardial CIR [13]. It is still unknown whether this pathway can act in the pathophysiology of ischemic stroke and whether it can regulate the pathophysiological process after CIR by regulating the oxidative stress pathway.

By constructing a CIR in vitro cell model, this study tried to clarify the role of the SNHG15-miR-141-SIRT1 pathway in CIR, to explore its role and mechanism on oxidative stress in OGD reoxygenated cells, and to assist the further treatment of CIR.

## 2. Experimental Methods

### 2.1. Bioinformatics Analysis

The primers for SNHG15 core connection points between obtained and SIRT1 were designed with StarBase (https://starbase.sysu.edu.cn/) and TargetScan (https//targetscan.org).

### 2.2. Luciferase Reporter Assay

SIRT1 3′ noncoding zones were synthesized, pCheck2 (Promega) was inserted downstream of the luciferase gene after annealing, and the Renilla site of the luciferase vector was reported. To introduce mutations, the sequence complementary (site: 5′ CUUUUGAAAUACAAAACCAGUGUUU-3′) to the binding sites of miR-141 in the 3′ UTR was replaced with site 5′-CUUGAAAUACAAAACCAGUGUUU-3′. The construction was confirmed by nucleotide sequencing. Wild-type or mutant plasmids, pCheck2 plasmids, and equal amounts of OGD-si-NC or miR-141 mimic plasmids were cotransfected into cells. A dual-luciferase reporter assay system was adopted to test the luciferase assay (Promega).

### 2.3. Cell Line and Cell Culture

SH-SY5Y cells were purchased from the cell bank of the Chinese Academy of Sciences (Shanghai). Cell-complete medium was DMEM (Sigma) supplemented with 10% fetal bovine serum (Invitrogen) and 100 U/mL penicillin/streptomycin (Sigma). The normal culture conditions were 10% fetal bovine serum and penicillin DMEM medium, cultured with 5% CO_2_ and 95% air at 37°C.

### 2.4. Oxygen-Glucose-Deprived Reoxygenation

When the SH-SY5Y cells reached 80% adherence, the culture medium was replaced by oxygen-free glucose-free balanced salt solution PBS and cultured with 5% CO_2_ and 95% air at 37°C for 15 h to simulate the OGD reoxygenation. Reoxygenation: the anaerobic glucose-free medium was replaced with a cell-complete medium cultured with 5% CO_2_ and 95% air at 37°C for 24 h.

### 2.5. Cellular Transfection

siRNA of miR-141 mimic and SNHG15 were purchased from GenePharma Company (Shanghai, China). Entrust the company to design and synthesize specific interference siRNA sequence against lncRNA SNHG15, miR-141 mimic sequence, and control siRNA sequence. The specific sequence is as follows: SNHG15 (Sense: 5′-UCA AAC UUG CUCAAUUAAGGU-3′, Anti-sence: 3′-CUUAAUUGAGCAAGUUUG AAA-5′) miR-141 mimic simulant (sense: 5′-UAA CAC UGU CUG GUA AAG AUG G-3′, Anti-sence: 5′-CAU CUU CCA GUA CAG UGU UGG A-3′). SNHG15 small interfering RNA (si-SNHG15 group) was transfected with Lipofectamine^TM^ 2000 liposome (Invitrogen, Karlsbad, CA, USA), and miR-141 mimics (miR-141 mimic group) were negative without a significant control group (si-con group); the transfection process was performed according to the instructions. After transfection for 6 h, the medium was replaced with the DMEM containing 10% fetal bovine serum. Then, the cells were cultured for another 48 h and placed in a constant temperature medium to collect cells for subsequent experiments.

### 2.6. RNA Extraction and qPCR Amplification

Cracking cells with TRIzol reagents, RNAs were extracted from SH-SY5Y cells in each group according to the instruction of the RNA extraction kit (Invitrogen, Shanghai, China). And then, synthetic cDNA was operated with the reverse transcription kit (Invitrogen, Shanghai, China). SYBR Green (Vazyme, Nanjing, China) was used for qPCR amplification at 95°C for 10 minutes, 95°C for 15 seconds, and 60°C for 1 minute, cycling for 40 times. qPCR primers of SNHG15 were as follows: SNHG15: forward: 5ʹ-CAACCATAGCGGTGCAACTGTGC-3ʹ; reverse: 5ʹGTACTGAACGTTGACCAAGTCGG-3ʹ; GAPDH primers: forward: 5′-CAGTGCCAGCCTCGTCTAT-3ʹ; reverse: 5ʹ-CTTCTGACACCTACCGGGGA-3′. The results were normalized according to the reference gene GAPDH of each parallel sample. In miRNA expression analysis, in RNAs (100 ng), reverse transcription was conducted with the TaqMan Advanced MicroRNA Assay kit (Applied Biosystems) and miRNA-specific primers. The primers (5′-CACTGTCTGGUAAAGA) of hsa-miR-141 for the detection with TaqMan MicroRNA were purchased from Applied Biosystems to calculate miR-141 relative expression. All experiments were repeated three times.

### 2.7. Western Blot Analysis

The proteins in cells of each group were extracted and centrifuged at 4 degrees and then added to the protein lysate for cell lysis with RIPA lysis buffer-combined protease inhibitor cocktail at a ratio of 99 : 1. After that, the total protein was quantified with the BCA method.

The proteins were transferred to the PVDF membrane by electrophoresis with 12% SDS polyacrylamide gel at 300mA2h and then sealed at room temperature with 5% skim milk sealant and TBST for 1 h. The primary antibodies were anti-SIRT1 antibody (diluted 1 : 2000, Abcam, catalog no. AB32441), anti-P65 antibody (diluted 1 : 1500, Abcam, catalog no. AB16502), anti-TNF-*α* antibody (diluted 1 : 500, Abcam, catalog no. AB6671), anti-IL-6 antibody (diluted 1 : 2000, Cell Signaling Technology, catalog no. 5216), iNOS antibody (diluted 1 : 2000, Santa Cruz Biotechnology, catalog no. SC-650), and GADPH antibody (1 : 5000, Abcam, catalog no. ab9485). All these antibodies were diluted with closed solution, incubated at room temperature for 1 h, and washed with PBS buffer 3 times for 5 min. The polyclonal goat anti-rabbit antibody 1 : 5000 (Cell Signaling Technology) diluted in the closed solution was used as the secondary antibody. Then, it was detected with ECL chemiluminescence reagent imaging (Amersham) and western blotting detection system (Millipore).

### 2.8. Statistical Analysis

Statistical data were analyzed by GraphPad Prism 7. Additional statistical analyses were performed with SPSS 20.0 (SPSS, Chicago, USA). PCR expression was statistically analyzed by Mann–Whitney *U*. The difference of miRNA and protein expression in vitro was detected with ANOVA. *P* value was calculated on both sides, and *P* < 0.05 was defined as statistically significant.

## 3. Results

### 3.1. SNHG15 Expression Increases in Oxygen-Glucose-Deprived Reoxygenation

The expression of SNHG15 and miR-141 in OGD reoxygenation was investigated.  Figure 1(a) shows the expressions of SNHG15 in OGD reoxygenation and normal cells detected by qRT-PCR, and Figure 1(b) shows the expressions of miR-141 in oxygen-glucose-deprivation reoxygenation and normal cells detected by qRT-PCR. The results suggest that, in cells in oxygen-glucose-deprivation reoxygenation, SNHG15 is higher than that of normal cells, and miR-141 is lower than that of normal cells. It indicates that SNHG15 and miR-141 play an important role in the pathophysiological mechanism of OGD reoxygenation in the nervous system.

### 3.2. SNHG15 Inhibits the miR-141 Expression of SH-SY5Y Cells in Oxygen-Glucose-Deprived Reoxygenation

SNHG15 miRNA was analyzed with StarBase and TargetScan to study the pathophysiological mechanism of SNHG15 in OGD reoxygenation. miR-141 is one of the miRNAs with the highest correlation with SNHG15 (FDR, *P* < 0.05). SIRT1 is the target gene of miR-141. In previous studies, miR-141 has been proved to play a role in OGD reoxygenation. Therefore, we speculate that SNHG15 may play a role in regulating miR-141 expression. To further test our hypothesis, we detected miR-141 expression in OGD-si-NC, miR-141 mimic, and SNHG15-siRNA groups with the qRT-PCR method and confirmed that miR-141 expression in both SNHG15-siRNA and miR-141-mimic groups was significantly higher than that in the OGD-si-NC group (Figure 2). The results showed that, in OGD reoxygenation, miR-141 expression increased after inhibiting SNHG15 expression. In conclusion, SNHG15 plays a role in the pathophysiological process of cells in OGD reoxygenation by inhibiting miR-141 expression.

### 3.3. miR-141 Negatively Regulates SNHG15 Expression

To see if miR-141 can also negatively regulate SNHG15, we examined SNHG15 expression in the miR-141 mimic group.  Figure 3 shows SNHG15 in OGD-si-NC, miR-141-mimic, and SNHG15-siRNA groups detected by qRT-PCR. The results showed that SNHG15 expression decreased in both SNHG15-siRNA and miR-141-mimic groups, suggesting that, as competitive endogenous RNA, miR-141 also negatively regulates SNHG15 expression.

### 3.4. SIRT1 May Be a Direct miR-141 Target

To identify miR-141 presumed mRNA targets, bioinformatics analysis was performed with two different microRNA target prediction tools, and several candidate targets were found. Among them, the SIRT1 mRNA 3′ UTR contained sequences complementary to miR-141 subsequences (Figure 4(a)). To verify whether SIRT1 is a direct miR-141 target, in the SIRT1 3′ noncoding zone, cells were cotransfected with three different plasmids, including wild-type or mutant plasmids, pCheck2 plasmids, and equivalent amounts of negative control or miR-141 mimic plasmids. Promega was used for luciferase detection. In transfected cells, a sustained decrease in luciferase activity was observed in miR-141 (Figure 4(b)). To further verify target specificity, we produced a 3′ UTR mutation (Figure 4(a)), where all the binding sites of miR-141 were destroyed by Q5 Site-Directed Mutagenesis Kit (NEB) that reduced 2 key nucleotides. NCs or miR-141 mimics were cotransfected with a mutant form of the 3′ UTR, significantly restoring luciferase activity (Figure 4(b)).

We further validated the effect of miR-141 on SIRT1 protein levels. miR-141 overexpression significantly decreased SIRT1 expression in SH-SY5Y cells (Figure 4(c)). Meanwhile, we verified that SNHG15 siRNA also reduced SIRT1 expression in SH-SY5Y cells (Figure 4(c)). To sum up, these data suggest that miR-141 inhibits SIRT1 expression in SH-SY5Y cells by directly targeting the 3′ UTR of cells, demonstrating that SNHG15 indirectly regulates SIRT1 expression by regulating miR-141 [3, 12].

### 3.5. miR-141 Regulates Oxidative Stress Pathways by Targeting SIRT1 Pathways

Recent studies have found that SIRT1 plays an important role in CIR by regulating the oxidative stress pathway [13]. Therefore, we sought to determine whether miR-141 plays a role in CIR by regulating the oxidative stress pathway through SIRT1. It is known that SIRT1 can inhibit the expression levels of p65, TNF-*α*, IL-1*β*, IL-6, iNOS, and other markers related to oxidative stress by regulating the NF-*κ*B pathway, thus playing a role in myocardial ischemia-reperfusion [14]. Therefore, to investigate whether SIRT1 affects oxidative stress pathways in CIR, the expression of oxidative stress markers was detected in the normal cell group and hypoxia-deficient group with western blotting expression patterns. As expected, SIRT1 overexpression led to the decrease of p65, TNF-*α*, IL-1*β*, IL-6, and iNOS levels (Figure 5). The expression of these oxidative stress signaling molecules was detected in SNHG15-siRNA and normal control hypoxia-deficient cells to further determine whether miR-141 regulates the oxidative stress signaling pathway by affecting SIRT1 expression. As shown in Figure 5, in miR-141-mimic and SNHG15-siRNA groups after miR-141 simulation, the overexpression of miR-141 significantly reduced the expression level of SIRT1, thereby increasing the expression level of oxidative stress-related molecules. To sum up, these data suggest that miR-141 regulates oxidative stress pathways by targeting SIRT1 expression.

## 4. Discussion

Recently, the role of lncRNAs in CIR has been confirmed by the literature as a potential target in the treatment of ischemic stroke [14]. SNHG15 expression increases in blood of patients with acute ischemic stroke, CIR rats, and cell models [10, 15], but the specific pathophysiological mechanism was not clear. In this study, the expressions of SNHG15, miR-141, and SIRT1 were investigated by constructing a neuronal CIR in vitro cell model and transfecting SNHG15 siRNA and miR-141 mimics, with the discussion on SNHG15, miR-141, and SIRT1 expressions. It is clear that the SNHG15-miR-141-SIRT1 pathway plays an important role in the pathophysiological process of CIR. After CIR, SNHG15 expression was upregulated, promoting the expression of its target gene SIRT1 by inhibiting miR-141 expression and thus promoting the expressions of relevant oxidative stress indicators, p65, TNF-*α*, IL-1*β*, IL-6, and iNOS, participating in the pathophysiological process of CIR by regulating the oxidative stress pathway.

In this study, SNHG15 could be a direct target for miR-141, regulating SIRT1 expression indirectly by regulating miR-141, speculating that lncRNA-miRNA-target genes can play important roles in the pathophysiological mechanism of OGD reoxygenation. Tian et al. [16] recently showed that SNHG8 could play a neuroprotective role in CIR as another lncRNA. SNHG8 overexpression could inhibit miR-425 expression and then reduce the expressions of TNF-*α* and other proinflammatory factors by regulating SIRT1 to reduce endothelial damage, which further confirmed the important role of SIRT1 in CIR. Zhou et al. [17] confirmed this conclusion that SNHG7 could also play a neuroprotective role in a rat ischemia-reperfusion model. SNHG7 overexpression inhibited miR-9 expression and reduced ROS production by regulating SIRT1 expressions. Consistent with the results of this study, SIRT1 might be a key gene for CIR, involving multiple lncRNAs and miRNAs in regulating SIRT1 expression, playing an important role in the pathophysiological mechanism of CIR.

In this study, SNHG15 expression increased in the OGD reoxygenation model, and it is speculated that it may act in OGD reoxygenation. SNHG15 was first thought to be tumor-related lncRNA, promoting the differentiation of tumor cells. SNHG15 expression in tumor cells was high. At the same time, it showed that limiting its expression might inhibit its invasion and metastasis in the tumor, and miR-141 acted as its sponge in the pathophysiological mechanism of CIR [18]. In recent years, studies have focused on the physiological mechanism of ischemic stroke and CIR. Deng et al. [10] showed that SNHG15 expression in human peripheral blood monocytes increased and positively correlated with the severity of the disease. Guo et al. [15] showed that SNHG15 expression increased in the rat middle cerebral artery blockage model and OGD N2a cell model, inhibiting SNHG15 expression which could alleviate neuronal death. All these findings were consistent with the conclusion in this study; we also confirmed that SNHG15 expression increased in OGD-SH-SY5Y cell models, indicating that SNHG15 played an important role in the pathophysiological mechanism of CIR.

In this study, inhibiting SNHG15 expression slowed down the oxidative stress response, leading to downregulation of the expressions of related inflammatory factors, assuming that SNHG15 plays a role in regulating oxidative stress. Many studies have also shown that oxidative stress plays an important role in the neuronal injury of ischemia-reperfusion and directly affects the prognosis of ischemic stroke. Wu et al. [19] showed that ROS production promotes CIR. Zhao et al. [20] also showed that protective oxidative stress can also slow neuronal apoptosis in CIR. Consistent with these conclusions, we found that the expression of restricted SNHG15 inhibited the expression of relevant oxidative stress factors in the OGD-SH-SY5Y cell model and, therefore, may further inhibit neuronal damage.

## 5. Conclusion

Numerous studies have shown that lncRNAs can act as miRNA endogenous sponges, regulating miRNA binding to target genes and thus participating in the relevant pathophysiological mechanism [4]. To further clarify the role of SNHG15 involved in neuroinflammation and oxidative stress in CIR cell models, we predicted the miRNA binding to it with bioinformatics software. It turned out that SNHG15 has miR-141-3p binding sites, which has also been confirmed in studies on other tumor diseases [18]. Zhou et al. [21] showed that miR-141 expression decreased in the PC12 CIR cell model, and miR-141 mimics could significantly improve cell damage after ischemia-reperfusion. However, inhibiting miR-141 expression can significantly aggravate cell damage. miR-141 could reduce the expressions of ROS, iNOS, and other indicators associated with oxidative stress and further slow down the injury of ischemia-reperfusion. Interestingly, Liu et al. [22] indicated that tumor necrosis factor-*α* (TNF-*α*) treatment could promote reperfusion injury and downregulate miR-141 expression. In our study, we found that SNHG15 siRNA could downregulate miR-141 expression. Meanwhile, miR-141 mimics could also promote SNHG15 expression, further promoting SNHG15-mediated pathophysiological processes. Therefore, we believe that SNHG15 can play a further role by regulating miR-141.

miRNA can regulate the expression of target genes by specifically binding to mRNA 3′ noncoding zones. For further clarification of the pathophysiological mechanism of miR-141 in CIR, we used the bioinformatics database for further prediction. It turned out that SIRT1 3′ noncoding zone may bind to miR-141 with specificity. Studies have shown that SIRT1 played a neuroprotective role in inhibiting apoptosis, slowing the inflammation, protecting mitochondrial function, and inhibiting oxidative stress in the pathophysiological mechanism of CIR [23]. Our findings confirmed this conclusion; SNHG15 siRNA may negatively regulate SIRT1 expression by promoting miR-141 expression and then increase the related proinflammatory factors and oxidative stress-related indicators such as TNF-*α*, IL-1*β*, and iNOS expressions. As mentioned earlier, there may be many lncRNAs and miRNAs that may play a role in the pathophysiological mechanism of CIR by regulating SIRT1 expression. However, their specific role may need further in vitro and in vivo experiments.

Overall, our study indicated that SNHG15 siRNA and miR-141 mimics reduce the expression of proinflammatory factors by interfering with the above pathways. Moreover, miR-141 mimics can also reduce SNHG15 expression and thus play a protective role. Our study showed that SNHG15 regulates neuroinflammation and oxidative stress through miR-141-mediated SIRT1 pathways and increases the expressions of proinflammatory factors and oxidative stress-related indicators, thus promoting neuronal damage in the pathophysiological process of CIR. This research explores its role and mechanism on oxidative stress in OGD reoxygenated cells to assist the further treatment of CIR. However, its specific role may need further in vitro and in vivo experiments. The lncRNAs and miRNAs' specific role still needs further in vitro and in vivo experiments.

## Figures and Tables

**Figure 1:** Expressions of SNHG15 and miR-141 in the oxygen-glucose-deprived reoxygenation model. (a) SNHG15 expression in the OGD group and control group of qRT-PCR analysis. (b) miR-141 expression in the OGD group and control group of qRT-PCR analysis, ^*∗*^*P* < 0.01.

**Figure 2:** Inhibition of SNHG15 on miR-141 expression in SH-SY5Y cells after OGD reoxygenation. Note: SH-SY5Y cells were transfected into OGD-si-NC, OGD-SNHG15-siRNA, and OGD-miR-141-mimic groups, respectively. miR-141 expression in the above three groups was detected by qRT-PCR, ^∗∗^*P* < 0.01.

**Figure 3:** Expression of SNHG15 and miR-141 in cells of each group. Note: SNHG15 expression in OGD-si-NC and OGD-miR-141-mimic groups was detected by qRT-PCR, ^∗∗^*P* < 0.01.

**Figure 4:** SIRT1 may be a hypothetical direct miR-141 target. (a) Luciferase report contains the miR-141 targeting sequences and mutated version of the SIRT1 3′ UTR wild type, including the site where the binding agent was altered (red). The luciferase reporter gene containing wild-type (Wt) or mutant SIRT1 3′ UTR (Mut) was cotransfected into SH-SY5Y cells by simulating NC or miR-141. (b) Luciferase activity was measured and normalized 72 h after transfection. (c) The protein level of transfected NC or miR-141 mimics and SNHG15-siRNA cells was detected by western blotting.

**Figure 5:** Regulation of miR-141 on oxidative stress pathways by targeting SIRT1. Note: three groups of hypoxia-deficient cells were transfected into OGD-si-NCs, miR-141-mimic, and SNHG15-siRNA groups. After transfection for 48 h, normal cultured cells and p65, TNF-*α*, IL-1*β*, IL-6, iNOS, and GADPH protein levels in three groups of normal cells treated with hypoxia and glucose deficiency were detected with western blot. Each band's strength was measured with ImageJ, normalized to GAPDH, and then normalized to NC-transfected cells.

## Data Availability

The datasets used and/or analyzed during the current study are available from the corresponding author upon reasonable request.
